The article "Adverse Pregnancy Outcomes Following Exposure to Biologics in Women With Crohn's Disease: A Systematic Review and Meta-Analysis" was retracted in 2022. Reasons: errors in the methods; unreliable results or conclusions; concerns about the data.

# Adverse Pregnancy Outcomes Following Exposure to Biologics in Women With Crohn's Disease: A Systematic Review and Meta-Analysis

**DOI:** 10.3389/fmed.2021.753088

**Published:** 2021-10-25

**Authors:** Han Wang, Fang Chen, Yue Hu, Mengdie Shen

**Affiliations:** ^1^Department of Gynecology and Obstetrics, Women's Hospital, School of Medicine, Zhejiang University, Hangzhou, China; ^2^Department of Gastroenterology, Hangzhou Red Cross Hospital, Hangzhou, China; ^3^Department of Gastroenterology, First Affiliated Hospital of Zhejiang Chinese Medical University, Hangzhou, China; ^4^Department of Internal Medicine, Women's Hospital, School of Medicine, Zhejiang University, Hangzhou, China

**Keywords:** Crohn's disease, adverse pregnancy outcomes, anti-TNF, anti-integrins, anti-interleukins

## Abstract

Crohn's disease is a chronic disease, which commonly affects women during their reproductive years. Poorly treated Crohn's disease is associated with adverse pregnancy outcomes. Biologics, a group of therapeutic drugs targeting inflammatory mediators including anti-TNF, anti-integrins and anti-interleukins, are increasingly used in pregnant women with Crohn's disease, exposing both the women and their fetuses to treatment-related complications. At present, it is unclear which biologics are more superior. This study performed a systematic review and meta-analysis to assess the risk of adverse pregnancy outcomes in women with Crohn's disease after exposure to biologics. Bibliographic databases were searched from inception to May 2021. The outcomes of interest were preterm delivery, low birth weight, spontaneous abortion, and congenital abnormalities. A total of 11 studies comprised of 1,875 pregnancies among women with Crohn's disease were included. Of these, 1,162 received biologics and 713 received non-biologic therapy. During the remission phase of the disease, the use of biological therapy increased the risk of adverse pregnancy outcomes, of which anti-integrins were associated with a higher incidence of adverse pregnancy outcomes than anti-TNF and anti-interleukins.

**Systematic Review Registration:** http://www.crd.york.ac.uk/PROSPERO, identifier: CRD42020191275.

## Introduction

Crohn's disease (CD) is a complex and life-long gastrointestinal inflammatory disease, characterized by gastrointestinal inflammation and several extraintestinal manifestations, leading to progressive intestinal injury and disability. The peak age of onset is in the second to the fourth decade that is consistent with the peak age for conception (1, 2).

Active CD during pregnancy is associated with an increased incidence of adverse pregnancy outcomes (APOs), including preterm delivery, low birth weight, spontaneous abortion, and congenital abnormalities (3–6). However, studies reporting on CD and birth outcomes may not always distinguish the impact of disease activity, drug use and CD severity on APOs (7). Therefore, it seems necessary for pregnant women with CD to receive medical specialist consultation to prevent the potential risk to the newborns. Increased awareness and understanding of the disease activity before and during pregnancy associated with the greatest risk of poor maternal and infant outcomes (8, 9) have encouraged more research to produce evidence and guidance on a treatment strategy that strives to achieve a balance between the risks of active disease and the risks of medications (10).

The article "Adverse Pregnancy Outcomes Following Exposure to Biologics in Women With Crohn's Disease: A Systematic Review and Meta-Analysis" was retracted in 2022. Reasons: errors in the methods; unreliable results or conclusions; concerns about the data.

A study has reported that patients with inflammatory bowel disease (IBD) may not have offspring because of their fear of adverse reproductive outcomes (11). Another study has also demonstrated that the frequency of voluntary childlessness among IBD patients is higher than that of the non-IBD control group (12). Therefore, the safety profile of biologics in pregnancy poses a major concern to pregnant women and their doctors. Through meta-analysis, this study aimed to quantify the risk of APOs in women with CD exposed to varying biologics, which would provide valuable evidence that guides optimal clinical decision-making.

## Methods

This systematic review was conducted using a pre-defined protocol and was reported based on the preferred reporting items of the systematic review and the statement of the systematic review meta-analysis (PRISMA) included in the meta-analysis of health care interventions (PROSPERO registration number: CRD42020191275).

### Search Strategy

Databases from Medline, PubMed, Web of Science, Embase and Cochrane Library were searched for relevant studies to evaluate the pregnancy outcomes of women with CD treated with biologics during pregnancy. All published studies and abstracts presented at the meetings were evaluated without any language restrictions. The reference list of the retrieved articles was also reviewed for more related research. The database search was conducted on 27th July 2020 and then updated on 27th May 2021.

### Study Selection

The title and abstract of each article were examined by three reviewers independently to eliminate duplication, comments, case reports and small case series (*n* < 10). The titles and abstracts of identified published articles were screened to exclude irrelevant studies. The full-text article was obtained and read if determined as eligible by at least one reviewer. Randomized controlled trials, observational and case-control studies were included in our analyses. Biologics that were market-authorized by either the U.S. Food and Drug Administration or European Medicines Agency were considered in our study. Any disagreements were discussed and resolved by consensus.

The article "Adverse Pregnancy Outcomes Following Exposure to Biologics in Women With Crohn's Disease: A Systematic Review and Meta-Analysis" was retracted in 2022. Reasons: errors in the methods; unreliable results or conclusions; concerns about the data.

The included studies met the following criteria: (1) Patients: pregnant women (age > 18 years) with CD in remission, who were exposed to biologics; (2) Intervention: biologics including anti-TNF agents (infliximab, adalimumab, certolizumab pegol, and golimumab), anti-integrin agents (vedolizumab, natalizumab), or anti-interleukin agents (ustekinumab, secukinumab, and tocilizumab) at any point during pregnancy; (3) Comparator: conventional therapy without biologics; (4) Outcomes: the overall rates of APOs were the key adverse outcomes, which comprised of preterm delivery, low birth weight, spontaneous abortion and congenital abnormalities.

Studies were excluded if: (1) trials that evaluated any drug treatment other than biologics; (2) trials of novel agents in development with only phase II RCT data (absence of phase III data); (3) studies in which pregnant women used biologics for an underlying disease other than CD; (4) trials that had an inadequate or absence of a control group, incomplete information on birth outcomes, provided data collected from other studies, or only evaluated differences between single treatment and combination therapy.

### Data Extraction and Quality Assessment

Full-text candidate articles were reviewed by three reviewers to determine the characteristics of the study population, the diseases treated, the drugs used, the number of sample populations, and the number of adverse outcomes. The authors of the articles were contacted if the data was not available immediately. Any disputes were resolved through discussion.

The Newcastle Ottawa Scale (NOS) was used to assess the quality of the included case-control and cohort studies (13). NOS is an evaluation tool for observational studies, which divides the grades of quality into three categories: study group selection, group comparability, and exposure (case-control study) or outcome (cohort study). Studies with a score of 5 or more on the 9-point scale were considered of high quality, while others were deemed as low quality. Any disagreements among reviewers were discussed and resolved by consensus.

### Statistical Analysis

The Mantel Haenszel method was used to calculate odds ratio (OR) and 95% confidence interval (CI). The choice of random or fixed models was based on the heterogeneity analysis (14). Heterogeneity was evaluated by *I*^2^ statistics, and fixed effect model was used for *I*^2^ < 50%; random effect model was used if *I*^2^ ≥ 50% (15). *I*^2^ > 50% indicated obvious heterogeneity in the study. Publication bias was assessed by examining for asymmetry in the funnel plot to determine the effectiveness of small studies (16). All statistical analyses were performed using RevMan (version 5.3.0, Copenhagen, Denmark).

The article "Adverse Pregnancy Outcomes Following Exposure to Biologics in Women With Crohn's Disease: A Systematic Review and Meta-Analysis" was retracted in 2022. Reasons: errors in the methods; unreliable results or conclusions; concerns about the data.

## Results

### Study Selection

The initial electronic and manual search yielded a total of 1,364 studies. Of these, 65 studies met our study criteria for further review, which revealed 21 case reports or small case series (*n* < 10), 19 retrospective studies and 25 prospective studies. Therefore, a total of 11 studies (three prospective, seven retrospective, and one prospective + retrospective studies) met the final selection criteria for inclusion in the meta-analysis (Figure 1).

**Figure 1:** Study flow diagram. Records identified by database searching and from gray literature. Sixty-five articles met the criteria for full-text review, with 11 finally included in the meta-analysis.

### Study Characteristics

The 11 eligible studies included a total of 1,875 cases. Of these, 972 pregnant women with CD were exposed to anti-TNFα therapy, 139 to anti-integrins therapy, 51 to anti-interleukins therapy and 713 were treated with non-biological therapy. The characteristics of the studies and pregnancy outcomes were outlined in Tables 1, 2, respectively.

**Table 1:** Characteristics of the studies included and the use of biologics during pregnancy.

**Study**	**Design**	**Pregnancies (*n*)**	**No. of pregnancies in the drug-exposed group**	**No. of pregnancies in the control group**	**Duration of exposure**	**Study quality**
Kammerlander et al. (17)	R	120	90 anti-TNF	30 BU	During the third trimester	✰✰✰✰✰✰✰
Zelinkova et al. (18)	P	50	25 anti-TNF (IFX+ADA)	25 BU	Discontinued the treatment at mean gestational week 22	✰✰✰✰✰✰✰
Lichtenstein et al. (19)	R	118	78 anti-TNF (IFX)	40 BU	At any time during pregnancy	✰✰✰✰✰
Wils et al. (20)	R	158	21 anti-integrins (VDZ) 27 anti-interleukins (UST) 60 anti-TNF (IFX)	50 BU	At any time within the 2 months prior to conception or during pregnancy	✰✰✰✰✰✰✰
Katz et al. (21)	R	164	82 anti-TNF (IFX)	82 BU	At any time within the 3 months prior to conception or during pregnancy	✰✰✰✰✰✰
Schnitzler et al. (22)	R	213	41 anti-integrins 48 anti-interleukins (UST) 72 anti-TNF (IFX+ADA)	52 BU	At any time within the 3 months prior to conception or during pregnancy	✰✰✰✰✰✰
Weber-Schoendorfer et al. (23)	P	222	27 anti-integrins 30 anti-interleukins (UST) 85 anti-TNF	80 BU	At any time during the first 12 weeks	✰✰✰✰✰✰✰
Clowse et al. (24)	P + R	396	53 anti-integrins 47 anti-interleukins 98 anti-TNF (CZP)	198 BU	At any time during pregnancy	✰✰✰✰✰✰✰
Moens et al. (25)	R	286	136 anti-TNF (IFX) 40 anti-integrins (VDZ) 24 anti-interleukins (UST)	86 BU	At any time within the 3 months prior to conception or during pregnancy	✰✰✰✰✰✰✰
Casanova et al. (26)	R	30	15 anti-TNF	15 BU	At any time within the 3 months prior to conception or during pregnancy	✰✰✰✰✰✰✰
de Lima et al. (27)	P	118	63 anti-TNF	55 BU	At any time during pregnancy	✰✰✰✰✰✰✰

*R, Retrospective; P, Prospective; BU, biologic unexposed*.

The article "Adverse Pregnancy Outcomes Following Exposure to Biologics in Women With Crohn's Disease: A Systematic Review and Meta-Analysis" was retracted in 2022. Reasons: errors in the methods; unreliable results or conclusions; concerns about the data.

**Table 2:** Pregnancy outcomes (proportion of adverse outcomes to the number of exposed pregnancies) of included studies.

**Outcomes group**	**Preterm delivery**				**Low birth weight**				**Spontaneous abortion**				**Congenital abnormalities**			
	**A**	**B**	**C**	**D**	**A**	**B**	**C**	**D**	**A**	**B**	**C**	**D**	**A**	**B**	**C**	**D**
Kammerlander et al. (17)	7/90			1/30	4/90			1/30								
Zelinkova et al. (18)									3/25			1/25	4/25			0/25
Lichtenstein et al. (19)	4/78			1/40					13/78			3/40	2/78			0/40
Wils et al. (20)	5/60	5/21	4/27	2/50	4/60	5/21	2/27	2/50	3/60	3/21	3/27	4/50	1/60	2/21	1/27	1/50
Katz et al. (21)									11/82			2/82				
Schnitzler et al. (22)	10/72	9/41	10/48	3/52	6/72	8/41	2/48	2/52	9/72	12/41	5/48	4/52	2/72	4/41	1/48	1/52
Weber-Schoendorfer et al. (23)	20/85	19/27	8/30	6/80	3/85	6/27	6/30	4/80	13/85			6/80	3/85			1/80
Clowse et al. (24)	5/98	6/53	3/47	4/198	2/98	3/53	2/47	4/198	10/98	9/53	4/47	10/198	3/98	5/53	1/47	2/198
Moens et al. (25)	14/136	10/40	4/24	10/86	16/136	12/40	4/24	7/86	18/136	6/40	4/24	9/86	4/136	3/40	1/24	2/86
Casanova et al. (26)	1/15			1/15	1/15			1/15	2/15			1/15	1/15			0/15
de Lima et al. (27)	5/63			2/55	6/63			2/55					2/63			1/55

*A, exposed to anti-TNF; B, exposed to anti-integrins; C, exposed to anti-interleukins; D, without biologics*.

### Adverse Pregnancy Outcomes

#### Preterm Delivery

There were nine studies that reported outcomes concerning preterm delivery that was defined as delivering at <37 weeks' gestation. When comparing pregnancies in women with CD exposed to biologics (*n* = 1,055) to those unexposed (*n* = 606), the OR of pooled crude rates of preterm deliveries was 2.87 (95% CI: 1.90, 4.32; *P* < 0.00001). No evidence of significant heterogeneity across the studies was identified (*P* = 0.40, *I*^2^ = 4%). Among the different biologics, the risk of preterm deliveries was significantly higher in the anti-integrins group than the anti-TNF group (OR: 3.26; 95% CI: 2.06, 5.18; *P* < 0.00001), with no significant heterogeneity observed among the studies (*P* = 0.30, *I*^2^ = 18%). When comparing between anti-interleukins and anti-TNF, there was no significant difference in the risk of preterm deliveries (OR: 1.48; 95% CI: 0.89, 2.47; *P* = 0.13) with no significant heterogeneity between the studies (*P* = 0.97, *I*^2^ = 0%). Further statistical comparison between anti-integrins and anti-interleukins revealed significantly higher risk of preterm deliveries among patients treated with anti-interleukins (OR: 2.07; 95% CI: 1.21, 3.55; *P* = 0.008), without significant heterogeneity between the studies (*P* = 0.23, *I*^2^ = 28%; Figure 2).

The article "Adverse Pregnancy Outcomes Following Exposure to Biologics in Women With Crohn's Disease: A Systematic Review and Meta-Analysis" was retracted in 2022. Reasons: errors in the methods; unreliable results or conclusions; concerns about the data.

**Figure 2:** Risk of preterm delivery in pregnant women treated with biologics for CD.

#### Low Birth Weight

There were eight studies reported on the outcomes concerning low birth weight among pregnant women with CD exposed to biologics. The OR of pooled crude rates of low birth weight was 2.26 (95% CI: 1.40, 3.65; *P* = 0.0009) when comparing those exposing to biologics (*n* = 953) to those unexposed (*n* = 566) and no significant heterogeneity was observed across studies (*P* = 1.00, *I*^2^ = 0%). Among the different biologics, the risk of low birth weight was significantly higher in patients treated with anti-integrins when compared with those treated with anti-TNF (OR: 3.58; 95% CI: 2.09, 6.14; *P* < 0.00001), and no significant heterogeneity was observed across studies (*P* = 0.82, *I*^2^ = 0%). When comparing anti-interleukins and anti-TNF, there was no significant difference in the risk of low birth weight (OR: 1.64; 95% CI: 0.86, 3.13; *P* = 0.13), with no significant heterogeneity between the studies (*P* = 0.19, *I*^2^ = 34%). Further comparison between anti-integrins and anti-interleukins revealed significantly higher risk of low birth weight among patients treated with anti-integrins (OR: 2.26; 95% CI: 1.18, 4.31; *P* = 0.01), without significant heterogeneity between the studies (*P* = 0.56, *I*^2^ = 0%; Figure 3).

**Figure 3:** Risk of low birth weight rate in pregnant women treated with biologics for CD.

### Spontaneous Abortion

There were nine studies reported on the outcomes concerning spontaneous abortion among pregnant women with CD exposed to biologics. The OR of pooled crude rates of spontaneous abortion was 2.13 (95% CI: 1.47, 3.10; *P* < 0.0001). When comparing those exposed to a biological agent (*n* = 952) to those unexposed (*n* = 628 and no evidence of heterogeneity observed across studies (*P* = 0.80, *I*^2^ = 0%). Among the different biologics, the risk of spontaneous abortion was significantly higher among patients treated with anti-integrins than those treated with anti-TNF (OR: 1.93; 95% CI: 1.14, 3.26; *P* = 0.01), and no significant heterogeneity was observed between the studies (*P* = 0.57, *I*^2^ = 0%). When comparing anti-interleukins and anti-TNF, there was no significant difference in the risk of spontaneous abortion (OR: 1.08; 95% CI: 0.57, 2.02; *P* = 0.82), with no observed significant heterogeneity between the studies (*P* = 0.71, *I*^2^ = 0%). Further comparison between anti-integrins and anti-interleukins demonstrated significantly higher risk of spontaneous abortion among patients treated with anti-integrins than those treated with anti-interleukins (OR: 1.96; 95% CI: 1.02, 3.78; *P* = 0.04), without significant heterogeneity across the studies (*P* = 0.47, *I*^2^ = 0%; Figure 4).

The article "Adverse Pregnancy Outcomes Following Exposure to Biologics in Women With Crohn's Disease: A Systematic Review and Meta-Analysis" was retracted in 2022. Reasons: errors in the methods; unreliable results or conclusions; concerns about the data.

**Figure 4:** Risk of spontaneous abortion in pregnant women treated with biologics for CD.

### Congenital Abnormality

There were nine studies reported on the outcomes concerning congenital abnormality outcomes among pregnant women with CD exposed to biologics. The OR of pooled crude rates of congenital abnormality was 2.91 (95% CI: 1.43, 5.94; *P* = 0.003), when comparing those exposed to biologics (*n* = 933) to those unexposed (*n* = 601), and no evidence of heterogeneity observed across the studies (*P* = 0.99, *I*^2^ = 0%). Among the different biologics, the risk of congenital abnormality was significantly higher among patients with anti-integrins than those treated with anti-TNF (OR: 3.48; 95% CI: 1.49, 8.11; *P* = 0.004), and no significant heterogeneity was observed between the studies (*P* = 0.95, *I*^2^ = 0%). When comparing between anti-interleukins and anti-TNF, there was no significant difference in the risk of congenital abnormality (OR: 1.05; 95% CI: 0.32, 3.46; *P* = 0.94) with no significant heterogeneity observed across the studies (*P* = 0.90, *I*^2^ = 0%). Further comparison of anti-integrins and anti-interleukins showed a significantly higher risk of congenital abnormality among patients treated with anti-integrins (OR: 3.52; 95% CI: 1.13, 10.97; *P* = 0.03), without significant heterogeneity between the studies (*P* = 0.92, *I*^2^ = 0%; Figure 5).

**Figure 5:** Risk of congenital abnormality in pregnant women treated with biologics for CD.

### Sensitivity Analysis

A “leave-one-out” sensitivity analysis showed that our analyses were robust and the elimination of every one included studies did not lead to any substantial change to our results.

## Discussion

To date, several treatments have been introduced for CD, including corticosteroids, 5-amino salicylate (5-ASA), biologics, immunosuppressive agents (28, 29), and antibiotics (30, 31), with probiotics (32) as supplemental therapy. Biologics such as anti-TNF, anti-integrins and anti-interleukins, are used widely to induce and maintain remission of CD (33). The treatment for pregnant IBD patients is especially challenging. Active IBD may deteriorate during pregnancy if without effective drug therapy. Studies have shown that among the pregnant women with active ulcerative colitis, 45% had deterioration of the disease, while one-third of those with active CD suffered worsening disease activity during pregnancy (34). When the disease is active at the time of pregnancy and during gestation, the risk of adverse pregnancy outcomes would be further increased (35, 36). To date, evidence is lacking on the safety of biologics for pregnant women with CD.

The article "Adverse Pregnancy Outcomes Following Exposure to Biologics in Women With Crohn's Disease: A Systematic Review and Meta-Analysis" was retracted in 2022. Reasons: errors in the methods; unreliable results or conclusions; concerns about the data.

Here, we conducted a meta-analysis to explore the risk of adverse pregnancy outcomes (preterm delivery, low birth weight, spontaneous abortion, and congenital abnormality) following the exposure to biologics (anti-TNF, anti-integrins, and anti-interleukins) in women with CD. A total of 1,162 pregnant women with CD treated with biologics were compared with 713 of those unexposed to biological therapy.

Our analyses revealed that the risks of preterm delivery, low birth weight, spontaneous abortion and congenital abnormality were all significantly increased in pregnant women exposed to biologics compared with those unexposed. Studies have shown that ~30–40% of women with IBD will have deterioration of their disease activity during pregnancy without medication (37). Also, a higher incidence of APOs in patients with IBD has been previously reported (38), whereby women with active IBD are at increased risk of preterm delivery, low birth weight and intrauterine growth restriction. However, the incidence of congenital malformations in the newborns of mothers with IBD is comparable with the general population (39). The study by de Lima et al. (27) has shown no increased risks of preterm delivery and low birth weight in pregnant women who continued anti-TNF treatment after 25 weeks of gestation when compared with those discontinuing treatment before 25 weeks of gestation. On the contrary, other studies have reported an increased incidence of preterm delivery and low birth weight in those treated with anti-TNF (3, 35, 40, 41).

Compared with the study by Casanova et al. (26) that only included 66 women who received anti-TNF therapy during pregnancy, our study has included a substantially greater sample size. Also, we have included anti-integrins and anti-interleukins therapy in the comparative analyses with anti-TNF. Our results revealed that compared with those using anti-TNF, the ORs of APOs in those treated with anti-integrins during pregnancy were 3.26 (95% CI: 2.06, 5.18) for preterm birth, 3.58 (95% CI: 2.09, 6.14) for low birth weight, 1.93 (95% CI: 1.14, 3.26) for spontaneous abortion, and 3.48 (95% CI: 1.49, 8.11) for congenital abnormality. Integrin plays a key role in mediating the binding of memory T lymphocytes to the mucosal of endothelial cell adhesion molecule 1 (MAdCAM-1), leading to infiltration into the gastrointestinal tract. Blocking this interaction can reduce the inflammatory cascades of IBD. From the therapeutic standpoint, a4 integrin is an ideal therapeutic target for IBD (42). Natalizumab, a humanized IgG4 monoclonal antibody, belongs to the FDA pregnancy Class C and has an unknown risk profile. Data on the safety of natalizumab usage during pregnancy and lactation are limited. In a small study (43), 164 patients with CD or multiple sclerosis were treated with natalizumab in the first 3 months of pregnancy, which showed no increased risk of congenital malformations. In accordance with the FDA, another anti-integrins drug, vedolizumab, can be used in pregnancy, despite lacking in studies on its fetotoxicity in humans and no long-term data are available (44). The placental metastasis is similar to other IgG drugs (infliximab, adalimumab), which increases linearly with the progress of the pregnancy. A prospective clinical study by Mahadevan et al. (45) has shown that among the 24 pregnant women treated with vedolizumab, there were 11 live births, 4 spontaneous abortions, 5 selective terminations of pregnancy, and 4 unrecorded outcomes.

The article "Adverse Pregnancy Outcomes Following Exposure to Biologics in Women With Crohn's Disease: A Systematic Review and Meta-Analysis" was retracted in 2022. Reasons: errors in the methods; unreliable results or conclusions; concerns about the data.

In our study, compared with those using anti-TNF, the ORs of adverse pregnancy outcomes in those treated with anti-interleukins during pregnancy were 1.48 (95% CI: 0.89, 2.47) for preterm birth, 1.64 (95% CI: 0.86 3.13) for low birth weight, 1.08 (95% CI: 0.57, 2.02) for spontaneous abortion, and 1.05 (95% CI: 0.32, 3.46) for congenital abnormality. A large meta-analysis comprised of 50,010 patients in 163 randomized clinical trials has revealed a similar safety profile between anti-interleukins therapy and anti-TNF agents (46). Consistently, our analyses also found no significant difference between anti-TNF and anti-interleukins in the risk of APOs. Due to the limited clinical application of anti-interleukins, all the anti-interleukin drugs included in our study were ustekinumab. The monoclonal antibody ustekinumab inhibits the p40 subunit of IL-12 and IL-23, which has been introduced for the treatment of CD (47). The specific blocking of IL-12 and IL-23 by ustekinumab is not only related to the pathophysiology of IBD but also to uterine physiology (48). IL-12 is an important cytokine in the process of uterine angiogenesis and vascular remodeling. During pregnancy, both high and low concentrations of IL-12 have been associated with early spontaneous abortion (48, 49). In addition, higher concentrations of IL-12 are associated with lower rates of fetuses that are small for gestational age in prematurely born infants (50). Therefore, ustekinumab can effectively impede the progression of CD and reduce the occurrence of adverse pregnancy outcomes, as evidenced in our analyses that when compared with anti-integrins, pregnant women treated with anti-interleukins had significantly lower risks of preterm delivery, low birth weight, spontaneous abortions, and congenital abnormalities.

The article "Adverse Pregnancy Outcomes Following Exposure to Biologics in Women With Crohn's Disease: A Systematic Review and Meta-Analysis" was retracted in 2022. Reasons: errors in the methods; unreliable results or conclusions; concerns about the data.

Most patients with CD have a long course of the disease, and conception is generally recommended when the disease is in remission. Our meta-analysis has revealed that during the remission phase of the CD, the use of biologics to maintain such remission is associated with a significantly higher risk of APOs. In particular, anti-integrins result in a higher incidence of APOs than anti-TNF and anti-interleukins. Therefore, the use of anti-integrins should be avoided while anti-TNF and anti-interleukins should be advocated for pregnant women CD.

## Data Availability Statement

The original contributions presented in the study are included in the article/supplementary material, further inquiries can be directed to the corresponding author/s.

## Author Contributions

FC and YH independently reviewed the title, abstract, or full text of all the identified articles. MS contacted to collect missing data or assess eligibility. Any disagreements regarding the eligibility of a study were resolved by mutual discussion (HW) or consultation with MS. All authors contributed to the article and approved the submitted version.

## Conflict of Interest

The authors declare that the research was conducted in the absence of any commercial or financial relationships that could be construed as a potential conflict of interest.

## Publisher's Note

All claims expressed in this article are solely those of the authors and do not necessarily represent those of their affiliated organizations, or those of the publisher, the editors and the reviewers. Any product that may be evaluated in this article, or claim that may be made by its manufacturer, is not guaranteed or endorsed by the publisher.

## References

[1] MottetC JuilleratP GonversJJ FroehlichF BurnandB VaderJP . Pregnancy and Crohn's disease. Digestion. (2005) 71:54–61. 10.1159/00008387415711051

[2] NguyenGC SeowCH MaxwellC HuangV LeungY JonesJ . The Toronto Consensus Statements for the management of inflammatory bowel disease in pregnancy. Gastroenterology. (2016) 150:734–57.e731. 10.1053/j.gastro.2015.12.00326688268

[3] de Lima-KaragiannisA Zelinkova-DetkovaZ van der WoudeCJ. The effects of active IBD during pregnancy in the era of novel IBD therapies. Am J Gastroenterol. (2016) 111:1305–12. 10.1038/ajg.2016.25427349339

[4] MahadevanU SandbornWJ LiDK HakimianS KaneS CorleyDA. Pregnancy outcomes in women with inflammatory bowel disease: a large community-based study from Northern California. Gastroenterology. (2007) 133:1106–12. 10.1053/j.gastro.2007.07.01917764676

The article "Adverse Pregnancy Outcomes Following Exposure to Biologics in Women With Crohn's Disease: A Systematic Review and Meta-Analysis" was retracted in 2022. Reasons: errors in the methods; unreliable results or conclusions; concerns about the data.

[5] MoserMA OkunNB MayesDC BaileyRJ. Crohn's disease, pregnancy, and birth weight. Am J Gastroenterol. (2000) 95:1021–6. 10.1111/j.1572-0241.2000.01852.x10763954

[6] NørgårdB HundborgHH JacobsenBA NielsenGL FonagerK. Disease activity in pregnant women with Crohn's disease and birth outcomes: a regional Danish cohort study. Am J Gastroenterol. (2007) 102:1947–54. 10.1111/j.1572-0241.2007.01355.x17573787

[7] NielsenOH LoftusEVJr. JessT. Safety of TNF-α inhibitors during IBD pregnancy: a systematic review. BMC Med. (2013) 11:174. 10.1186/1741-7015-11-17423902720PMC3734216

[8] StephanssonO LarssonH PedersenL KielerH GranathF LudvigssonJF . Crohn's disease is a risk factor for preterm birth. Clin Gastroenterol Hepatol. (2010) 8:509–515. 10.1016/j.cgh.2010.02.01420202483

[9] ØstensenM CetinI. Autoimmune connective tissue diseases. Best Pract Res Clin Obstet Gynaecol. (2015) 29:658–70. 10.1016/j.bpobgyn.2015.03.00325891380

[10] KavanaughA CushJJ AhmedMS BermasBL ChakravartyE ChambersC . Proceedings from the American College of Rheumatology Reproductive Health Summit: the management of fertility, pregnancy, and lactation in women with autoimmune and systemic inflammatory diseases. Arthritis Care Res (Hoboken). (2015) 67:313–25. 10.1002/acr.2251625385050

[11] MountifieldR BamptonP ProsserR MullerK AndrewsJM. Fear and fertility in inflammatory bowel disease: a mismatch of perception and reality affects family planning decisions. Inflamm Bowel Dis. (2009) 15:720–5. 10.1002/ibd.2083919067431

[12] MarriSR AhnC BuchmanAL. Voluntary childlessness is increased in women with inflammatory bowel disease. Inflamm Bowel Dis. (2007) 13:591–9. 10.1002/ibd.2008217206690

[13] StangA. Critical evaluation of the Newcastle-Ottawa scale for the assessment of the quality of nonrandomized studies in meta-analyses. Eur J Epidemiol. (2010) 25:603–5. 10.1007/s10654-010-9491-z20652370

[14] DerSimonianR LairdN. Meta-analysis in clinical trials. Control Clin Trials. (1986) 7:177–88. 10.1016/0197-2456(86)90046-23802833

[15] StroupDF BerlinJA MortonSC OlkinI WilliamsonGD RennieD . Meta-analysis of observational studies in epidemiology: a proposal for reporting. Meta-analysis Of Observational Studies in Epidemiology (MOOSE) group. JAMA. (2000) 283:2008–12. 10.1001/jama.283.15.200810789670

[16] HigginsJP ThompsonSG DeeksJJ AltmanDG. Measuring inconsistency in meta-analyses. BMJ. (2003) 327:557–60. 10.1136/bmj.327.7414.55712958120PMC192859

[17] KammerlanderH NielsenJ KnudsenT KjeldsenJ FriedmanS NørgårdBM. Anti-TNF-α use during the third trimester of pregnancy in women with moderate-severe inflammatory bowel disease and the risk of preterm birth and low birth weight. Inflamm Bowel Dis. (2017) 23:1916–23. 10.1097/MIB.000000000000123428858070

The article "Adverse Pregnancy Outcomes Following Exposure to Biologics in Women With Crohn's Disease: A Systematic Review and Meta-Analysis" was retracted in 2022. Reasons: errors in the methods; unreliable results or conclusions; concerns about the data.

[18] ZelinkovaZ van der EntC BruinKF van BaalenO VermeulenHG SmalbraakHJ . Effects of discontinuing anti-tumor necrosis factor therapy during pregnancy on the course of inflammatory bowel disease and neonatal exposure. Clin Gastroenterol Hepatol. (2013) 11:318–21. 10.1016/j.cgh.2012.10.02423103819

[19] LichtensteinGR FeaganBG MahadevanU SalzbergBA LangholffW MorganJG . Pregnancy outcomes reported during the 13-year TREAT registry: a descriptive report. Am J Gastroenterol. (2018) 113:1678–88. 10.1038/s41395-018-0202-930022113

[20] WilsP SeksikP StefanescuC NanceyS AllezM Pineton de ChambrunG . Safety of ustekinumab or vedolizumab in pregnant inflammatory bowel disease patients: a multicentre cohort study. Aliment Pharmacol Ther. (2021) 53:460–70. 10.1111/apt.1619233345331

[21] KatzJA AntoniC KeenanGF SmithDE JacobsSJ LichtensteinGR. Outcome of pregnancy in women receiving infliximab for the treatment of Crohn's disease and rheumatoid arthritis. Am J Gastroenterol. (2004) 99:2385–92. 10.1111/j.1572-0241.2004.30186.x15571587

[22] SchnitzlerF FidderH FerranteM BalletV NomanM Van AsscheG . Outcome of pregnancy in women with inflammatory bowel disease treated with antitumor necrosis factor therapy. Inflamm Bowel Dis. (2011) 17:1846–54. 10.1002/ibd.2158321830263

[23] Weber-SchoendorferC OppermannM WackerE BernardN BeghinD Cuppers-MaarschalkerweerdB . Pregnancy outcome after TNF-α inhibitor therapy during the first trimester: a prospective multicentre cohort study. Br J Clin Pharmacol. (2015) 80:727–39. 10.1111/bcp.1264225808588PMC4594709

[24] ClowseMEB ScheuerleAE ChambersC AfzaliA KimballAB CushJJ . Pregnancy outcomes after exposure to certolizumab pegol: updated results from a pharmacovigilance safety database. Arthritis Rheumatol. (2018) 70:1399–407. 10.1002/art.4050829623679PMC6174965

[25] MoensA van der WoudeCJ JulsgaardM HumbletE SheridanJ BaumgartDC . Pregnancy outcomes in inflammatory bowel disease patients treated with vedolizumab, anti-TNF or conventional therapy: results of the European CONCEIVE study. Aliment Pharmacol Ther. (2020) 51:129–38. 10.1111/apt.1553931692017

[26] CasanovaMJ ChaparroM DomènechE Barreiro-de AcostaM BermejoF IglesiasE . Safety of thiopurines and anti-TNF-α drugs during pregnancy in patients with inflammatory bowel disease. Am J Gastroenterol. (2013) 108:433–40. 10.1038/ajg.2012.43023318480

[27] de LimaA ZelinkovaZ van der EntC SteegersEA van der WoudeCJ. Tailored anti-TNF therapy during pregnancy in patients with IBD: maternal and fetal safety. Gut. (2016) 65:1261–8. 10.1136/gutjnl-2015-30932125966992

The article "Adverse Pregnancy Outcomes Following Exposure to Biologics in Women With Crohn's Disease: A Systematic Review and Meta-Analysis" was retracted in 2022. Reasons: errors in the methods; unreliable results or conclusions; concerns about the data.

[28] RahimiR NikfarS AbdollahiM. Do anti-tumor necrosis factors induce response and remission in patients with acute refractory Crohn's disease? A systematic meta-analysis of controlled clinical trials. Biomed Pharmacother. (2007) 61:75–80. 10.1016/j.biopha.2006.06.02217184965

[29] NikfarS MirfazaelianH AbdollahiM. Efficacy and tolerability of immunoregulators and antibiotics in fistulizing Crohn's disease: a systematic review and meta-analysis of placebo-controlled trials. Curr Pharm Des. (2010) 16:3684–98. 10.2174/13816121079407923621143147

[30] FeaganBG SandbornWJ HassS NieckoT WhiteJ. Health-related quality of life during natalizumab maintenance therapy for Crohn's disease. Am J Gastroenterol. (2007) 102:2737–46. 10.1111/j.1572-0241.2007.01508.x18042106

[31] LoftusEV FeaganBG ColombelJF RubinDT WuEQ YuAP . Effects of adalimumab maintenance therapy on health-related quality of life of patients with Crohn's disease: patient-reported outcomes of the CHARM trial. Am J Gastroenterol. (2008) 103:3132–41. 10.1111/j.1572-0241.2008.02175.x18853973

[32] ElahiB NikfarS DerakhshaniS VafaieM AbdollahiM. On the benefit of probiotics in the management of pouchitis in patients underwent ileal pouch anal anastomosis: a meta-analysis of controlled clinical trials. Dig Dis Sci. (2008) 53:1278–84. 10.1007/s10620-007-0006-z17940902

[33] ScheinfeldN. Off-label uses and side effects of infliximab. J Drugs Dermatol. (2004) 3:273–84. 15176162

[34] KatzJA PoreG. Inflammatory bowel disease and pregnancy. Inflamm Bowel Dis. (2001) 7:146–57. 10.1097/00054725-200105000-0001111383588

[35] KammerlanderH NielsenJ KjeldsenJ KnudsenT FriedmanS NørgårdB. The effect of disease activity on birth outcomes in a nationwide cohort of women with moderate to severe inflammatory bowel disease. Inflamm Bowel Dis. (2017) 23:1011–8. 10.1097/MIB.000000000000110228346274

[36] O'TooleA NwanneO TomlinsonT. Inflammatory bowel disease increases risk of adverse pregnancy outcomes: a meta-analysis. Dig Dis Sci. (2015) 60:2750–61. 10.1007/s10620-015-3677-x26070523

[37] FergusonCB Mahsud-DornanS PattersonRN. Inflammatory bowel disease in pregnancy. Bmj. (2008) 337:a427. 10.1136/bmj.39566.681458.BE18599468PMC2483894

[38] DominitzJA YoungJC BoykoEJ. Outcomes of infants born to mothers with inflammatory bowel disease: a population-based cohort study. Am J Gastroenterol. (2002) 97:641–8. 10.1111/j.1572-0241.2002.05543.x11926208

[39] KwanLY MahadevanU. Inflammatory bowel disease and pregnancy: an update. Expert Rev Clin Immunol. (2010) 6:643–57. 10.1586/eci.10.3520594137

The article "Adverse Pregnancy Outcomes Following Exposure to Biologics in Women With Crohn's Disease: A Systematic Review and Meta-Analysis" was retracted in 2022. Reasons: errors in the methods; unreliable results or conclusions; concerns about the data.

[40] SeirafiM de VroeyB AmiotA SeksikP RoblinX AllezM . Factors associated with pregnancy outcome in anti-TNF treated women with inflammatory bowel disease. Aliment Pharmacol Ther. (2014) 40:363–73. 10.1111/apt.1283324980270

[41] BrömsG GranathF LinderM StephanssonO ElmbergM KielerH. Birth outcomes in women with inflammatory bowel disease: effects of disease activity and drug exposure. Inflamm Bowel Dis. (2014) 20:1091–8. 10.1097/MIB.000000000000006024810137

[42] XavierRJ PodolskyDK. Unravelling the pathogenesis of inflammatory bowel disease. Nature. (2007) 448:427–34. 10.1038/nature0600517653185

[43] NazarethM CristianoL KoojimansM. Natalizumab use during pregnancy. Am J Gastroenterol. (2008) 103:S449.

[44] MahadevanU MatroR. Care of the pregnant patient with inflammatory bowel disease. Obstet Gynecol. (2015) 126:401–12. 10.1097/AOG.000000000000097826241432

[45] MahadevanU VermeireS LaschK AbhyankarB BhayatF BlakeA . Vedolizumab exposure in pregnancy: outcomes from clinical studies in inflammatory bowel disease. Aliment Pharmacol Ther. (2017) 45:941–50. 10.1111/apt.1396028169436

[46] SinghJA WellsGA ChristensenR Tanjong GhogomuE MaxwellL MacdonaldJK . Adverse effects of biologics: a network meta-analysis and Cochrane overview. Cochrane Database Syst Rev. (2011) 2011:CD008794. 10.1002/14651858.CD008794.pub221328309PMC7173749

[47] FeaganBG SandbornWJ GasinkC JacobsteinD LangY FriedmanJR . Ustekinumab as induction and maintenance therapy for Crohn's disease. N Engl J Med. (2016) 375:1946–60. 10.1056/NEJMoa160277327959607

[48] Lédée-BatailleN DubanchetS Coulomb-L'hermineA Durand-GasselinI FrydmanR ChaouatG. A new role for natural killer cells, interleukin (IL)-12, and IL-18 in repeated implantation failure after in vitro fertilization. Fertil Steril. (2004) 81:59–65. 10.1016/j.fertnstert.2003.06.00714711545

[49] WieringaJW DriessenGJ Van Der WoudeCJ. Pregnant women with inflammatory bowel disease: the effects of biologicals on pregnancy, outcome of infants, and the developing immune system. Expert Rev Gastroenterol Hepatol. (2018) 12:811–8. 10.1080/17474124.2018.149682029972674

[50] NetaGI von EhrensteinOS GoldmanLR LumK SundaramR AndrewsW . Umbilical cord serum cytokine levels and risks of small-for-gestational-age and preterm birth. Am J Epidemiol. (2010) 171:859–67. 10.1093/aje/kwq02820348155PMC2877445

